The article "Application Value of Elbow Pressing Method Combined with Zhongtong Ling Application in Children with Swelling and Pain after Operation of Supracondylar Fracture of the Humerus" was retracted in 2023. Reasons: unreliable results or conclusions; lack of ethics approval or compliance; concerns about the data; concerns about the peer review.

# Application Value of Elbow Pressing Method Combined with Zhongtong Ling Application in Children with Swelling and Pain after Operation of Supracondylar Fracture of the Humerus

**DOI:** 10.1155/2022/8594443

**Published:** 2022-08-23

**Authors:** Liyi Qiu, Youren Wang, Xiaoyu Wang

**Affiliations:** ^1^Beijing Massage Hospital, Beijing 100035, China; ^2^Special Clinic, Beijing Massage Hospital, Beijing 100035, China; ^3^Tuina Department, Beijing Chaoyang Integrated Traditional Chinese and Western Medicine Emergency Rescue Center, Beijing 100035, China

## Abstract

In order to improve the treatment effect of supracondylar fracture of the humerus, the application value of elbow press combined with Zhongtong Ling paste in postoperative swelling and pain in children with supracondylar fracture of the humerus is analyzed. 82 children with humeral condylar fracture undergoing surgery in our hospital from March 2019 to May 2020 are selected and divided into the control group and research group according to the symptoms of soreness. The VAS score is used to observe and compare the pain degree before intervention (T1), 1 month after intervention (T2), and 3 months after intervention (T3).The Kaplan–Meier survival curve is obtained to observe the recurrence rate of swelling and pain in the two groups. Besides, the satisfaction scale designed by our hospital is employed to evaluate parents' satisfaction with the treatment. The application of Zhongtong Ling ointment combined with elbow compression can effectively improve the curative effect, improve children's pain, and promote rehabilitation in the treatment of postoperative swelling and pain of supracondylar fracture of the humerus in children.

## 1. Introduction

Supracondylar fracture of the humerus refers to the fracture above the medial and lateral condyles of the distal humerus. Humeral supracondylar fractures are mostly caused by indirect violence, and most of them occur in sports injuries, life injuries, and traffic accidents [1]. According to the fracture displacement, the straightening type can be divided into the straightening ulnar deviation and the straightening radial deviation [2]. The characteristics of extended supracondylar fracture of the humerus are as follows: the fracture line is located at or above the level of the olecranon fossa in the lower segment of the humerus, the direction of fracture is from anterior lower to posterior upper, the fracture is angled forward, and the distal end is displaced backward. The fracture line of flexion humeral supracondylar fracture can be transverse, the fracture is angled backward, and the distal fracture end moves forward or has no obvious displacement [3]. Supracondylar fracture of the humerus is more common in elbow joint injury in children, accounting for 72%, and children are mostly 5–8 years old [4]. From the clinical manifestation, the elbow joint of the patient was unable to move locally after injury, and the swelling was obvious. There is a bone triangle relationship at the elbow, indicating no dislocation. The elbow is in the half bend position, and the elbow socket is full. Sometimes the fracture end of the humerus can be touched in the cubital fossa [5]. If it is impossible to make a careful examination due to swelling and pain, X-ray should be taken quickly to determine the fracture and displacement. Children cannot move freely after an elbow fracture, which will also swell and affect their health, which is not conducive to physical development [6]. At present, closed reduction and Kirschner wire internal fixation is the main method of clinical treatment, which has the characteristics of no obvious scar, fast recovery, small trauma, and so on. When the supracondylar fracture of the humerus is not treated properly, Volkmann ischemic muscle contracture or cubitus varus deformity may be easily caused. However, there are abundant blood vessels and nerves near the elbow joint, so soft tissue swelling and pain often occur during the operation, affecting the postoperative recovery. Although various treatment methods have been improved, which have significantly reduced Volkmann ischemic muscle contracture, cubitus varus deformity continues to occur and the incidence is still high, which must be paid attention to during treatment. After long term research, it is found that traditional Chinese medicine has a good performance in alleviating postoperative swelling and pain. Especially in elbow exercise therapy, doctors put their fingers or palms on a certain acupoint or part of the patient's joints to make active or passive corresponding movements [7] to achieve the purpose of combing muscles and tendons, restoring joint position, anti-inflammatory and pain relief. Our hospital has achieved an ideal curative effect in the treatment of traumatic diseases. Based on clinical experience, this study explored the treatment of swelling and pain after the humeral supracondylar fracture in children with elbow joint movement combined with Zhongtong Ling.

The rest of the paper is organized as follows: Section 2 discusses related studies, and Section 3 presents the information and methodology. In Section 4, the results and analysis are given. The conclusions are presented in Section 5.

## 2. Related Work

After operation for the supracondylar fracture of the humerus in children, swelling of limbs may occur due to inflammatory reaction, abnormal local microcirculation, and exudation [8]. In addition, pain symptoms may occur due to stimulation and compression of the peripheral nerve. The occurrence of postoperative swelling and pain will reduce the comfort and compliance of children, which is not conducive to postoperative recovery. Traditional intervention methods included acupuncture, cold compress, and intravenous drip of 20% mannitol, and sodium aescinate, but the effect will be affected by children's tolerability [9].

Traditional Chinese medicine believes that after a fracture, due to broken bones and tendons, the meridians are damaged, blood overflows outside the veins, and bad blood stays inside, which is blood stasis [10]. Because Qi moved with blood, blood stasis blocks Qi and airflow was not smooth, resulting in abnormal operation of Qi and blood. Moreover, blood stasis did not disperse, and blood stasis swelled in skin muscles and muscles [11]. When external force caused the limb fracture, the vein of the affected limb was involved, and Qi stagnation and blood stasis occurred. Therefore, a large amount of blood accumulates in the affected area, and swelling of varying degrees will occur. The lack of Qi and blood was the root cause of pain [12]. After the fracture, the limbs were injured, thereby causing damage to the meridians, and the blood flow was not smooth, resulting in swelling of the wound. According to the Golden Book of medical science, the circulation of blood and Qi in the human body was slightly stagnant [13]. Acupoint massage had the functions of dredging meridians, activating blood circulation and removing blood stasis, and supplementing Qi and detumescence. These findings provided a theoretical basis for the elbow joint exercise therapy for the supracondylar fracture of the humerus in children. Meridian massage and acupoint application were common in traditional Chinese medicine treatment. The principle of the meridian massage was to massage some acupoints, so as to dredge the meridians and reduce the incidence rate of diseases [14]. The principle of the acupoint application was to apply drugs and acupoints together, which can adjust the body and relax tendons [15]. Furthermore, it can effectively promote blood circulation and fully reflect the effect of drugs. In terms of the ingredients of externally applied traditional Chinese medicine, Radix Paeoniae Alba and Radix Angelicae dahuricae have the functions of dredging menstruation, relieving pain, and activating blood circulation. Angelica sinensis, Ligusticum chuanxiong, safflower, and frankincense had the functions of activating blood circulation, dredging collaterals, and reducing swelling and pain [16].

Exercise therapy was an important technology in massage. It was a massage treatment method characterized by doctor-patient cooperation and the combination of movement and rest [17]. Under the guidance of the basic theory of traditional Chinese medicine, especially the meridian theory and the five-body theory, specific manipulation was used to act on the corresponding parts or acupoints of the human body. It can enable patients to carry out active or passive limb movement or respiratory movement, so as to achieve the purpose of preventing and treating diseases. Elbow massage can effectively alleviate local muscle adhesion, smooth local muscle fibers, and play an anti-inflammatory and analgesic role [18]. Acupoint meridian's movement combined with Zhongtong Ling application can play a faster detumescence role in the treatment of pediatric fractures because traditional Chinese medicine can promote blood circulation, remove blood stasis, and quickly relieve pain. In addition, it can also promote the formation of callus and the recovery of limb function in patients [19, 20]. Elbow pressing activity therapy is a massage method that stimulates specific acupoints and performs physical activities to make the meridians more smooth, and achieve the effects of reducing swelling and itching, promoting blood circulation and removing blood stasis [21, 22]. The combination of elbow push stimulation and drug penetration therapy has good therapeutic effects. It can reduce the severe pain in time and help to achieve better results. In this study, Zhongtong Ling application combined with elbow massage can quickly alleviate swelling and pain symptoms, promote the formation of callus, and lay the foundation for the recovery of elbow function. Research showed that elbow joint movement combined with Zhongtong Ling patch can not only quickly and effectively alleviate children's swelling and pain but also improve the satisfaction of children's family members.

## 3. Information and Methodology

### 3.1. General Information

82 children with a humeral condylar fracture undergoing surgery in our hospital from March 2019 to May 2020 are enrolled in this study. The children are divided into the reference group (*n* = 41): age range 2–13 years, mean (7.02 ± 1.31) years, and the ratio of female to male patients 17 : 24 and the study group (*n* = 41): age range 3–12 years, mean (6.89 ± 1.56) years, and the female to male ratio 18 : 23. The basic data of children are compared, and the difference is very small (*P* > 0.05), reaching the comparative study standard, see Table 1 for details.

Inclusion criteria are as follows:

1. Have high therapeutic compliance and communication ability
2. The drug used at the age of years has no allergic symptoms
3. The clinical data and general information are complete
4. There should be swelling and pain

Exclusion criteria are as follows:

1. The wound is damaged
2. Mental diseases
3. Ability of self-management is poor and cannot be treated as required
4. Disconnect during treatment

The detailed comparison of baseline data is illustrated in Table 1.

### 3.2. Method

#### 3.2.1. Treatment Mode

The children in the reference group are treated with traditional Chinese medicine Zhongtong Ling application at the same time in routine treatment. The prescription is composed of Angelica dahurica 3 g, *Glycyrrhiza* 3 g, Clematis 3 g, Honghua 3 g, Chuan Dong 3 g, Danggui 5 g, olibanum 6 g, Herba speranskia tuberculate 6 g, and Jitongpi 6 g. After the cream is prepared, it is applied at acupoints such as Yanggu, Houxi, Jiangliao, Waiguan, Yangxi, and Hegu.

The treatment basis of the study group is combined with elbow massage intervention in the reference group. The basic manipulation is as follows: (1) The child is in the sitting position or supine position, and the doctor is on the affected side. (2) The rolling method, kneading method, dipping method, or one-finger Zen method are applied 3∼5 times on the radial side of the forearm. (3) We take the radial side of the forearm 3∼5 times and click Quchi, Shou Sanli, Chize, and Shaohai acupoint. (4) We click Yangxi and Zhouliao acupoints. (5) We click the Jianzhen acupoint upward, lift the twist Waiguan acupoint, and click the tennis elbow point (0.5 inches on the pillow acupoint, that is, 1 inch on the second and third metacarpophalangeal joints on the back of the hand). (6) This line is about 2 cm long in the radial side of Chize acupoint, and the doctor used this line as a method of kneading.

Next, the local pressing method is adopted as follows: (1) Elbow flexion and extension pressing method: Child sitting position. The doctor is located on the affected side, with the thumb of one hand pressing the curved cistern and pain point of the elbow on the affected side, and the other hand holding the wrist of the affected side to make the elbow joint flex and extend passively for 3∼5 times. (2) The elbow rotation toggle method is applied. The doctor is located on the affected side, with one hand holding the curved cistern of the elbow on the affected side or the point of pain in the three limbs of the hand, and the other hand holding the wrist on the affected side to make the elbow joint rotate passively inside and outside for 3∼5 times so that the child can tolerate it.

#### 3.2.2. Observation Indicators

The observation indicators are as follows: (1) Rehabilitation effect. The postoperative swelling recovery of children in two groups is evaluated. (2) Effectiveness. The degree of swelling symptom relief is 30–70%. (3) Significant effect. The degree of swelling symptom relief is 71–95%. (4) Recovered rate. Swelling symptoms relieved to over 95% or completely subdued swelling.

#### 3.2.3. VAS Scale

This scale is mainly used to assess the pain degree of children. The specific operation is to draw a straight line with a length of 10 cm on the paper, with a header marked with 0 points, representing no pain. The other header is 10 points, representing extreme pain, and the patient is asked to make a mark on the straight line according to self-feeling, representing the pain at this time. A score of less than or equal to 3 indicates mild pain that can be tolerated. A 4∼ score of six indicates that pain has affected sleep but is still tolerable. A score of 7 or more indicates that pain is unbearable and affects daily life.

#### 3.2.4. Self-Made Satisfaction Scale

The scale is self-made by the hospital and is scored 4, 3, 2, 1, and 0, respectively, according to very satisfactory, satisfactory, general, unsatisfactory, and very unsatisfactory. The main contents include recovery speed, pain degree, the influence of daily living ability, and self-reported feelings of children.

### 3.3. Statistical Analysis

SPSS 25.0 statistical software is used for data analysis. If the measurement data are subject to normal distribution and homogeneity of variance after a normal test, they are expressed by mean + standard deviation, and the matched sample *t* is used for the test within the group; variance comparison is used between groups. Repeated measures analysis of variance (ANOVA) is used for multiple time points within the group, and the spherical test is performed. For counting data, the percentage is used for descriptive statistical analysis, and the x2 test is used. All the above data showed significant differences at *P* < 0.05.

## 4. Results and Analysis

### 4.1. Comparison of the Effect of Swelling Recovery of Children in Each Group

Compared with the reference group, the overall response rate of children in the study group is higher, and the difference is statistically significant (*P* < 0.05), as shown in Table 2.

### 4.2. Comparison of the Pain Degree of Children in Each Group at Different Time Points

There is no significant difference in the degree of pain between the two groups before treatment (*P* > 0.05). There is a significant difference in VAS scores between the two groups (*P* < 0.05), as shown in Table 3 and Figure 1. The marks “*∗*” and “#” represent the comparison of the result with T1 and T2, respectively. The symbol “a,” “b,” and “c,” respectively, indicate that if the letters in the group are common, *P* > 0.05.

### 4.3. Recurrence Rate of Swelling and Pain in Children within Three Months

The Kaplan–Meier survival curve showed that the recurrence rate of four children in the study group is significantly smaller than that in the reference group (11 cases), accounting for 9.8% and 26.8%. The difference between the two groups is statistically significant (*x*^2^ = 0.998, *P*=0.046), as shown in Figure 2.

### 4.4. Comparison of the Satisfaction of the Family Members of the Two Groups

The results showed that the mean scores of the parents' satisfaction with the treatment regimen in the study group are significantly higher than those in the reference group (*P* < 0.05), as shown in Table 4 and Figure 3.

## 5. Conclusion

In this study, the application value of elbow press combined with Zhongtong Ling paste in postoperative swelling and pain in children with the supracondylar fracture of the humerus is analyzed. 82 children with a humeral condylar fracture undergoing surgery in our hospital from March 2019 to May 2020 are selected and divided into the control group and research group according to the symptoms of soreness. The VAS score is used to observe and compare the pain degree before intervention (T1), 1 month after intervention (T2), and 3 months after intervention (T3). The children with postoperative swelling and pain of the supracondylar fracture of the humerus are treated by routine Zhuantong Ling application, and at the same time, elbow massage is carried out according to the moving method, which could alleviate postoperative pain of children, promote rehabilitation, and is worthy of clinical practice.

## Figures and Tables

**Figure 1:** Difference in VAS scores between two groups.

**Figure 2:** Kaplan–Meier survival curve of the recurrence rate of swelling and pain in two groups.

**Figure 3:** Comparison of parent satisfaction in two groups.

**Table 1:** Comparison of baseline data.

	Study group (*N* = 41)	Control group (*N* = 41)	*t/x* ^2^	*P*
Age (Years)	7.02 ± 1.31	6.89 ± 1.56	0.409	0.684
Gender			0.050	0.823
Man	24 (58.54%)	23 (56.10%)		
Woman	17 (41.46%)	18 (43.90%)		
BMI (kg/m)	15.52 ± 2.03	15.42 ± 2.12	0.218	0.828

**Table 2:** Comparison of clinical treatment effects between two groups of children (*n*, %).

Grouping	Number of cases	Heal	Significant effect	Effective	Invalid	Overall response rate
Study group	41	12 (29.27)	19 (46.34)	8 (19.51)	2 (4.88)	39 (95.12)
Reference group	41	9 (21.95)	13 (31.71)	10 (24.39)	9 (21.95)	32 (78.05)
*x * ^2^						5.145
*P*						0.023

**Table 3:** Difference in VAS scores between two groups.

Group	T1	T2	T3	*F*	*P*
Study group (*n* = 41)	8.52 ± 1.43	5.66 ± 2.12 ^*∗*^	2.12 ± 0.17 ^*∗#*^	3.843	0.004
Reference group (*n* = 41)	9.25 ± 2.07	7.88 ± 1.61 ^*∗*^	5.64 ± 1.91 ^*∗#*^	4.455	0.035
*t*	−1.858	−5.340	−11.754		
*P*	0.067	<0.001	<0.001		

**Table 4:** Difference between the two groups of parents' satisfaction with the treatment scheme.

Group	Satisfaction score
Study group (*n* = 41)	18.52 ± 2.44
Reference group (*n* = 41)	12.91 ± 4.49
*t*	7.029
*P*	<0.001

## Data Availability

The simulation experiment data used to support the findings of this study are available from the corresponding author upon request.
